The article "A Study of Two-Way Short- and Long-Term Memory Network Intelligent Computing IoT Model-Assisted Home Education Attention Mechanism" was published in 2021. Journal: Comput Intell Neurosci.

# A Study of Two-Way Short- and Long-Term Memory Network Intelligent Computing IoT Model-Assisted Home Education Attention Mechanism

**DOI:** 10.1155/2021/3587884

**Published:** 2021-12-21

**Authors:** Suling Ma

**Affiliations:** Lishui University, Lishui, Zhejiang 323000, China

## Abstract

This paper analyzes and collates the research on traditional homeschooling attention mechanism and homeschooling attention mechanism based on two-way short- and long-term memory network intelligent computing IoT model and finds the superiority of two-way short- and long-term memory network intelligent computing IoT model. The two-way short- and long-term memory network intelligent computing IoT model is improved and an improved deep neural network intelligent computing IoT is proposed, and the improved method is verified based on discrete signal homeschooling classification experiments, followed by focusing on the application research of the two-way short- and long-term memory network intelligent computing IoT model-assisted homeschooling attention mechanism. Learning based on neural network, human behavior recognition method combining spatiotemporal networks, a homeschooling method integrating bidirectional short- and long-term memory networks and attention mechanisms is designed. The visual attention mechanism is used to add weight information to the deep visual features extracted by the convolutional neural network, and a new feature sequence incorporating salient attention weights is output. This feature sequence is then decoded using an IndRNN independent recurrent neural network to finally classify and decide on the homeschooling category. Experiments on the UCF101 dataset demonstrate that the incorporation of the attention mechanism can improve the ability of the network to classify. The attention mechanism can help the intelligent computing IoT model discover key features, and the self-attention mechanism can effectively capture the internal features of homeschooling and optimize the feature vector. We propose the strategy of combining the self-attention mechanism with a bidirectional short- and long-term memory network to solve the family education classification problem and experimentally verify that the intelligent computing IoT model combined with the self-attention mechanism can more easily capture the interdependent features in family education, which can effectively solve the family education problem and further improve the family education classification accuracy.

## 1. Introduction

With the continuous improvement of the material level, the state's investment in family education has gradually increased, and people's demand for scientific family education concepts has become more and more urgent. The establishment of the National Family Education Association has provided favorable theoretical support for the development of family business in our country. Research articles and monographs on family education have emerged as the times require. Its research involves multiple perspectives and can be divided into three categories: one is popular science: reading materials; the second category is popular reading materials with a story complex; the third category is theoretical research works [1]. Family education is emotional, and an important feature of family education is that it is contagious. Family education is the communication between parents and children and the positive or negative influence of parents' words, actions, and behavior on girls [2]. Parents are their children's role models and life mentors in the process of growth. In the current situation, deep learning has achieved an overwhelming victory in the fields of speech recognition, natural language processing, and homeschooling recognition, which has greatly contributed to the changes in other fields [3]. Applying deep learning to home education data processing can replace the traditional method of manually labeling data to achieve real-time processing of each piece of data received, which greatly saves the time of manual labeling and can effectively improve the efficiency of home education analysis [4].

The article "A Study of Two-Way Short- and Long-Term Memory Network Intelligent Computing IoT Model-Assisted Home Education Attention Mechanism" was published in 2021. Journal: Comput Intell Neurosci.

Internet of Things technology, as a new generation of information technology, is an important third type of information technology after computer technology and Internet technology, and it is also a new wave ushered in by the information industry. The emergence of the Internet of Things regulates the communication and interactive control of information between people and things and things and things, which are integrated with the Internet through various wireless or wired networks. The attention model is applied to the analysis of the attention mechanism of family education, and the attention mechanism is added to the family education framework to weigh the input features to measure the importance of each feature to the current recognition, focusing on the important features and ignoring the unimportant features. The attention model is applied to family education attention mechanism analysis to extract feature information [5]. The self-attention mechanism, as a special kind of attention mechanism, is introduced into the homeschooling classification task to be able to learn the word dependencies within sentences and capture the internal structure of homeschooling. Therefore, this paper explores the current technical points in the field of family education analysis from the practical needs of family education analysis and seeks to find an efficient and accurate family education analysis method based on deep learning technology and self-attention mechanism. With the rapid development of deep learning technology, neural network models represented by convolutional neural networks and recurrent neural networks have obtained remarkable research results in the field of natural language processing, and people use these models for family education data analysis to obtain certain practical value [6].

The article "A Study of Two-Way Short- and Long-Term Memory Network Intelligent Computing IoT Model-Assisted Home Education Attention Mechanism" was published in 2021. Journal: Comput Intell Neurosci.

While neural networks have so many advantages, they also inevitably have some drawbacks. The structure of neural networks and the corresponding training methods need to be specified in advance, which requires extensive design experience. The reasonable design of the network structure is very important to the accuracy of the modeling, the network structure is not reasonable to a large extent affecting the subsequent application of the network, and only the model structure is selected properly to make it play the proper value [7]. The selection of the initial value of the network also has an impact on the modeling, which is directly related to the convergence process of the weight training. If the initial value is not selected appropriately, it will prolong the training time, reduce the network accuracy, and weaken the generalization ability.  Section 1 is the introduction. This section introduces the research background and significance of the paper and also outlines the organization of the paper.  Section 2 is the related work. The direction and value of this paper's research are analyzed in light of the current research status at home and abroad.  Section 3 is a study on the mechanism of home education attention based on two-way short- and long-term memory network intelligent computing IoT model assistance. This section uses a combination of a two-way long- and short-term memory network and intelligent computing IoT model to classify the supervised education dataset, and the algorithm can greatly improve the classification accuracy of home education compared with the traditional method.  Section 4 is the result analysis. This section analyzes the data for the classified family education dataset using a bidirectional short- and long-term memory network intelligent computing IoT model and attention mechanism techniques to achieve good family education classification results.  Section 5 is the conclusion. This section systematically summarizes the research content of the thesis, analyzes the shortcomings, and provides an outlook on the next improvement direction.

## 2. Current Status of Research

The basis of computational intelligence can also be understood as the continuous evolution of structures. Since the birth of intelligent computing, its powerful intelligence, robustness, and self-adaptability have attracted the attention of many researchers, and great breakthroughs have been made in both theoretical research and practical applications of algorithms [8]. Kolomvatsos and Anagnostopoulos proposed a simple two-way short- and long-term memory network intelligent computing IoT algorithm for recommendation classification or nonrecommendation, which predicts the outcome by the average semantic of specific phrases in home education, with an average accuracy of 74% in the final experiment [9]. George and Santra proposed a combination of natural language processing and fuzzy logic techniques for analyzing homeschool content in homeschooling, and the experiments showed a very good correspondence between sentiment sets and human judgments of homeschool content [10]. Mollah et al. obtained rich emotional features by fusing machine learning methods and multiple rules and integrated them into the basic feature model, which improved the classification effect in the microblog sentiment classification experiment. Semantic rules are integrated into the support vector machine model to complete sentiment analysis tasks [11]. Experiments have verified that the support vector machine model combined with semantic rules is more effective in sentiment classification tasks [12]. The neural network can process the sequence information of text data and calculate and sort the influence of the input object on the final classification result. According to the sorting result, the words with strong emotional tendencies are assigned higher weights to reduce the loss of emotional information.

The article "A Study of Two-Way Short- and Long-Term Memory Network Intelligent Computing IoT Model-Assisted Home Education Attention Mechanism" was published in 2021. Journal: Comput Intell Neurosci.

While neural networks have so many advantages, they inevitably have some shortcomings. The structure of the neural network and the corresponding training method need to be specified in advance, which requires us to have rich design experience [13]. Zhang et al. obtained C&W models by deep neural network training and applied them to processing tasks such as home education labeling and home education classification and achieved good results [14]. Ge et al. used convolutional neural networks for homeschooling analysis tasks and conducted comparative experiments on seven datasets by combining convolutional kernels of different sizes with maximum pooling to demonstrate the effectiveness of single-layer CNNs in homeschooling classification tasks [15]. Wang and Ashwini proposed several recurrent neural networks such as RNN, MRNN, and RNTN, among which the RNTN model used syntactic analysis trees to obtain [16]. To imitate the sentence structure, McCormack et al. used a tree LSTM model to model family education and obtained excellent results in the family education classification task, which was input to the LSTM according to the temporal relationship to construct a CNN-LSTM model and apply it to the family education analysis task [17]. The content of family education should be rich and diversified, not limited to the traditional family education content, but diversified mainly in that the content of family education should involve all aspects of moral, intellectual, physical, aesthetic, and social development [18].

At present, how to apply the two-way short- and long-term memory network intelligent computing IoT model and attention mechanism to home education polarity analysis is still in the research stage, and the research goal of this thesis is to construct an efficient and accurate home education classification method. Based on this, the main research contents and innovations of this research work include the following three aspects. The loss function in deep neural networks has a significant influence on model training overfitting. To make the home education binary classification model more effective in overfitting the samples with prediction errors [19], local linearization in time limits the applicability of the proposed method in the discrete-time domain and impairs its prediction accuracy under strong nonlinear conditions. In the testing process, the idea of online learning was used for reference, and artificial judgment and relearning mechanisms were added to further improve the accuracy of network labeling. Experiments show that the automatic labeling algorithm can effectively improve the efficiency and accuracy of thermal measurement data analysis. According to the ranking results, higher weights are assigned to the categories with stronger family education tendencies to reduce the loss of family education information. Accordingly, this paper designs a bidirectional short- and long-term memory network intelligent computing IoT model and verifies the effectiveness of the model through quantitative and qualitative experiments on different homeschooling datasets [20].

## 3. Research on the Mechanism of Home Education Attention Based on Two-Way Short- and Long-Term Memory Network Intelligent Computing IoT Model Assistance

### 3.1. Feature Extraction of Family Education Attention Mechanism Based on Two-Way Long- and Short-Term Memory Network

In this paper, we combine BN-Inception with IndRNN to propose a deep learning human behavior recognition model with fused spatiotemporal networks. The spatial flow network deals with homeschooling attention mechanism features, which are mainly used to capture features with strong differentiation for action understanding; the temporal flow network deals with continuous optical flow features, which are used to learn effective action features. This makes full use of the temporal and spatial dimensional information of the data, increases the depth of the network while reducing the complexity of the network, and finally achieves the purpose of improving the accuracy of behavior recognition. The feature model of the homeschooling attention mechanism based on the bidirectional short- and long-term memory network proposed in this paper is shown in Figure 1.

The article "A Study of Two-Way Short- and Long-Term Memory Network Intelligent Computing IoT Model-Assisted Home Education Attention Mechanism" was published in 2021. Journal: Comput Intell Neurosci.

Since the obtained family education data also records the starting position of the effective value in the whole curve, firstly, the whole heat flow curve is divided into three sections according to the starting position, including the invalid data section before the effective data section, the valid heat flow segment, and the invalid data segment after the valid data segment. After that, divide the two large invalid data segments into several segments. The specific method is to use the length of the valid segment as the length of the data segment, and then from the beginning of the invalid data segment, follow the sliding window in steps of 0.9 times the length. The method moves backward in turn, thus dividing the invalid data segment into multiple segments. This article adopts the variation equation (1) of the family education problem. The first term is the regularization term to obtain a smooth displacement field.

(1) $$\begin{array}{c} \text{variation}=\min\left(\int \left|\forall {\left(x_{1}\right)}^{2}+\forall {\left(x_{2}\right)}^{2}\right|\text{d}\varpi \int \left|H_{1}\left(x+u\left(x\right)\right)-H_{0}{\left(x\right)}^{2}\right|\varpi \right). \end{array}$$

The mean intensity difference between pixels is therefore used as the homeschooling similarity score. Thus, the target parallax map is the minimum of equation (2). The optical flow algorithm uses the H_1_ parametrization to solve for minimization of the error function and minimization of the regular term of the target homeschool. Given two homeschooling frames H_0_ and H_1_, the objective is to find the parallax map such that the error function and the canonical term of homeschooling are minimized simultaneously, where the first term is the fidelity of the homeschooling data and the second term is the a priori canonical term. *β* denotes the correlation coefficient between the fidelity and the canonical term.

(2) $$\begin{array}{c} G\left(x\right)=\int \left[\alpha \beta \left(H_{0}\left(x\right)-H_{1}\left(x+u\left(x\right)\right)\right)+\varpi \left(x_{1},x_{2}\right)\right]\text{d}x. \end{array}$$

The effect of education depends on the consistency of the influence of the school and the family. If there is no such consistency, then the school's teaching and education process collapse like a paper house. School teachers communicate with parents in time through home visits and parent meetings. The weight coefficient of each subsection is learned through the visual attention mechanism, and the probability distribution of each subsection is finally fused, and the IndRNN cyclic neural network is input for sequence learning. Finally, the results of IndRNN are used in the behavior prediction of the family education level.

The article "A Study of Two-Way Short- and Long-Term Memory Network Intelligent Computing IoT Model-Assisted Home Education Attention Mechanism" was published in 2021. Journal: Comput Intell Neurosci.

The bidirectional short- and long-term memory network considers the temporal dimensional association of the convolutional neural network feature sequences, and the pooling operation only produces feature vectors that keep the temporal order constant. We assume that the feature sequences extracted by the spatial and temporal flow networks are *X* = (*x*_1_, *x*_2_,…,*x*_T_), so the independent recurrent neural network (IndRNN) computes a sequence of hidden vectors with N neurons at each moment *t H* = (*h*_1_, *h*_2_,…,*h*_T_) and the output vector sequence *f*(*t*) = (*y*_1_, *y*_2_,…,*y*_T_), satisfying equation (3), where A denotes the weight coefficient from the previously hidden layer to the current hidden layer, and *A*(*h*_0_) denotes the weight coefficient from the hidden layer to the output layer, *β* denotes the deviation coefficient, and *h*(*t*) denotes the hidden vector of the *n*th neural unit at moment *t*.

(3) $$\begin{array}{c} \left\{\begin{array}{c} n=\left[1,2,3,\ldots ,N\right],\\ f\left(t\right)=A\left(h_{0}\right)*h_{1}+\beta \left(t\right),\\ h\left(t\right)=H\left(A\left(h_{i}\right)\infty *y\left(t\right)+A\left(h_{h}\right)*y\left(t-1\right)+\beta \left(t\right)\right). \end{array}\right. \end{array}$$

The computation of the bidirectional LSTM model in the hidden layer is the same as that of the hidden layer of the LSTM and is passed between the same layers and the parameters are shared. Therefore, let the parameters of forwarding propagation be *V* and the parameters of backward propagation be *U*. Then the forward propagation formula of the bidirectional LSTM is as follows:

(4) $$\begin{array}{c} \left\{\begin{array}{c} \text{Lstm}\left(h_{t}\right)=B\left(t\right)*\;\sin\left(h\left(\zeta \left(t\right)\right)\right),\\ \text{Lstm}\left(h_{t}^{*}\right)=B^{*}\left(t\right)*\;\sin\left(h\left(\zeta {\left(t\right)}^{*}\right)\right). \end{array}\right. \end{array}$$

After the forward propagation of the network is finished, the output is done as a Softmax operation to obtain the predicted value yˆ with the true label value *y* to calculate the loss function. The experiment uses cross-entropy as the loss function, so the derivation of the backpropagation process of the bidirectional LSTM is the same as the derivation of the backpropagation process of the LSTM, as in the following equation:

(5) $$\begin{array}{c} \frac{\text{d}\left(f\left(t\right)\right)}{\text{d}W}=\beta *\left(1-\beta \right)*\left(\beta \left(t\right)++\zeta \left(t\right)+B^{*}*f\left(t\right)+W*M{\left(t-1\right)}^{*}\right). \end{array}$$

The article "A Study of Two-Way Short- and Long-Term Memory Network Intelligent Computing IoT Model-Assisted Home Education Attention Mechanism" was published in 2021. Journal: Comput Intell Neurosci.

### 3.2. Intelligent Computing IoT Model Construction

The practical activities in the virtual-real integration environment are different from the traditional practical activities, which put forward higher requirements on teaching, environment, model, and process. Based on the characteristics of the comprehensive practical activities course and the current situation research, this study, combined with the Internet, the characteristics of the IoT, and other information technology, made adaptable modifications based on Cooper's experiential cycle learning circle and summarized the comprehensive practical activities teaching based on experiential learning theory. The five elements of the model are precursor learning, practical inquiry, extension and expansion, observation and reflection, and communication and evaluation. The calculation process of the self-attentive mechanism is divided into three steps. Step one is to calculate the similarity between an element and a keyword, the second step is to normalize the original score, and finally, the weighted sum of the weighted values according to the obtained weighting coefficients is used to find the value of self-attentive for the element. The keyword is denoted by *K*, the function is denoted by *F*, the query is denoted by *Q*, the data source is denoted by *S*, the similarity is denoted by Sam, the attention value is denoted by *A*, and the value of the weight coefficient is denoted by *V*. Here *Q* = *K* = *V*; when home education is entered, self-attention is calculated once.

Different functions and computer mechanisms are introduced according to the query and keywords, and then the similarity between the two is calculated, and the intelligent calculation of the IoT calculation formula is shown in the following equation:

(6) $$\begin{array}{c} \text{Sam}\left(Q,K\right)=\sum_{i=1}^{N}MLP\left(Q,K_{i}\right). \end{array}$$

A calculation method similar to Softmax is introduced to convert the score obtained in the previous step to obtain the weight coefficient *ai*. The calculation formula is formula (7). Determine a confidence threshold above the threshold is a valid data segment, and below the threshold is an invalid data segment. Input the multiple pictures finally obtained in the third step into the trained convolutional neural network again to obtain the confidence level of each picture. These confidences are compared with the previous confidence thresholds, and two demarcation segments are obtained, which are lower than the threshold and higher than the threshold.

(7) $$\begin{array}{c} f\left(x\right)Fax\left(\text{Sam}\left(x\right)\right)=\frac{x^{\text{Sam}\left(i\right)}}{\sum_{i=1}^{N}x^{\text{Sam}\left(i\right)}}. \end{array}$$

When the input sequence *n* is smaller than the representation dimension *d*, the time complexity self-attention mechanism of each layer is the smallest. When *n* is relatively large, one solution is a restricted self-attention mechanism; that is, each word is not calculated with all words, but only with restricted *r* words. The force mechanism and the convolutional neural network can be well paralleled and do not rely on the previous calculation, which is better than the cyclic neural network; in terms of long-distance dependence, the self-attention mechanism can combine any two sentences in a sentence through a calculation result. Words are connected, so the long-distance dependence feature is greatly shortened, and its maximum path length is 1, which can capture long-distance dependence. The text data within a certain sliding window is converted into a fixed-length vector B” by the Softmax function, and then the feature data is fed into a linear SVM classifier for training and outputting the sentiment classification results, which is calculated by equation (8), where C denotes the training error of the SVM classifier, W and H denote the final obtained weight matrix and bias value, respectively, and *L* denotes the loss function.

(8) $$\begin{array}{c} \left\{\begin{array}{c} B^{\prime \prime }=\text{Soft }\max\left(w*B\prime +\beta \right),\\ C\left(W,M\right)=\frac{\sum_{i=1}^{M}\sum_{j=1}^{N}H_{ij}\left(B^{\prime \prime }\right)}{M*N}+\alpha *Y\left(W\right). \end{array}\right. \end{array}$$

When the neural network model is trained, the selection and setting of parameters is a very important aspect, and the training results will be very different when different parameters are selected, and the parameter settings of the model in this section are shown in Table 1.

The article "A Study of Two-Way Short- and Long-Term Memory Network Intelligent Computing IoT Model-Assisted Home Education Attention Mechanism" was published in 2021. Journal: Comput Intell Neurosci.

The cross-entropy loss function, also called the logarithmic loss function, is designed for the performance comparison of classification models and can be divided into dichotomous cross-entropy and multiclassification cross-entropy according to the difference of whether the classification model is dichotomous or multiclassification. It has the mathematical expression of the following equation:

(9) $$\begin{array}{c} G\left(x\right)=\sum_{i=1}^{N}\sum_{j=1}^{N}g\left(x_{i}\right)+\log\;Y\left(x_{i}\right),\;x_{i}=y\left(i\right)+j. \end{array}$$

Traversing the entire dataset to compute the loss function once and update the gradient of each parameter, this method is called batch gradient descent, and the parameters are updated using equation (10). *G*(*x*) is the value of the *k*th parameter at *x* iterations, *H*(*x*) is the first-order partial differential of the error function corresponding to that parameter, and *ρ* is the step size (learning rate), which indicates the size of the step, which determines the length of each step along the negative direction of the gradient, and a current optimal value is generally obtained by the linear search, which increases the computational effort and affects the performance of the model and does not support online learning.

(10) $$\begin{array}{c} G\left(x+1\right)=G\left(x\right)-\rho *\forall G\left(x\right)*H\left(x\right). \end{array}$$

### 3.3. Classification Evaluation of Family Education Attention Mechanism

When a predictive classifier is used to process binary sample data, we usually classify the sample data into two categories: Positive (Positive) and Negative (Negative). When the family education sample is classified as positive, it means the classification is correct, so we call it True Positive (PT) or true positive; when the positive family education sample is classified into the negative family education sample, it means the classification is wrong. Call it False Negative (NF) or false negative. Similarly, when dealing with negative sample data, if the classifier classifies the negative sample data into a negative class, the negative sample data is correctly classified, and we call it True Negative (NT) or true negative; if the negative sample data is classified into positive class, it means the classification is wrong, and we call it False Positive (FP) or false positive. The prediction effect is evaluated according to the value of the metric in the following equation:

(11) $$\begin{array}{c} \left\{\begin{array}{c} \text{NS}=\frac{\text{PT}}{\text{NF}+\text{PT}}*100\%,\\ \text{PS}=\frac{\text{NT}}{\text{NT}+\text{PF}}*100\%,\\ \begin{array}{c} \text{ACC}=\frac{\text{NT}+\text{PT}}{\text{TOTAL}}*100\%,\\ \text{TOTAL}=\text{PF}+\text{PT}+\text{NF}+\text{NT,} \end{array}\\ \text{MCC}=\frac{\left(\text{PT}*\text{NT}\right)-\left(\text{PF}*\text{NF}\right)}{\sum \sqrt{\left(\text{PT}+\text{PF}\right)*\left(\text{PT}+\text{NF}\right)*\left(\text{NT}+\text{PF}\right)*\left(\text{NT}+\text{FNF}\right)}}*100\%, \end{array}\right. \end{array}$$

where NS is the sensitivity metric for classification, and the magnitude of the NS value can be observed to understand how well positive samples are classified as positive samples. PS is the classifier specificity metric, which calculates the percentage of negative sample data that are classified as negative classes. Acc is the accuracy rate, and the metric reflects the percentage of positive and negative samples that are both correctly classified at the time of classification. MCC value, also known as the MCC correlation coefficient metric, reflects the Sn and PS metrics between the equilibrium degree of NS and PS is shown by the above equation; when the difference between these two indicators is smaller, MCC is larger.

The article "A Study of Two-Way Short- and Long-Term Memory Network Intelligent Computing IoT Model-Assisted Home Education Attention Mechanism" was published in 2021. Journal: Comput Intell Neurosci.

In the evaluation process of the attention mechanism of family education, there are soft evaluation aspects such as the humanization of model construction and design and the innovation of model construction. Therefore, the evaluation method of this article adopts very good, good, average, poor, and very poor. Describe the related problems, realize the primary level evaluation, and then use fuzzy mathematics to make the fuzzy information numerical, to carry out quantitative analysis and evaluation.

When multiple features are included in the training model, the dimensionality of the mixed feature vector may become very large, and due to the presence of more random information and noise in the uneven initial features, it will hurt the training model, and usually to solve such problems a feature selection tool such as F-score [25] can be used to select the most effective features. Therefore, we also call F-score a metric to identify features between different categories based on the F-score value, and the larger the F-score value, the stronger the differentiation of such features between different categories. The expressions for calculating F-score are shown in the following equation:

(12) $$\begin{array}{c} F\left(\text{score}\right)=\frac{\sum_{i=1}^{M}\left(x_{i}^{+}-x_{i}^{-}\right)}{m^{+}-1}+\frac{\sum_{i=1}^{M}\left(x_{i}^{+}-x_{i}^{-}\right)}{m^{-}-1}. \end{array}$$

In some of the discrete classifiers or two-classified classifiers we use, their classification decisions (Y or N) at each output can be represented by a single point in the ROC space, and all the points in the threshold interval converge into a curve, the ROC curve, so we can use this ROC curve to represent this threshold interval. Further, we express the performance depicted by the ROC curve, the AUC value, with the formula as in equation (13), while the specific diagnostic descriptions are shown in Table 2.

(13) $$\begin{array}{c} \text{Value}\left(\text{AUC}\right)=\int_{-\propto }^{+\propto }\left(NS\left(x\right)*\text{FPR}\left(x\right)\right)\text{d}x. \end{array}$$

In equation (13), *x* denotes the cutoff value of classification prediction probability and FPR denotes the percentage of negative samples being predicted as positive samples for the following equation:

(14) $$\begin{array}{c} \text{FPR}=\frac{\text{PF}}{\text{NT}+\text{PF}}. \end{array}$$

The article "A Study of Two-Way Short- and Long-Term Memory Network Intelligent Computing IoT Model-Assisted Home Education Attention Mechanism" was published in 2021. Journal: Comput Intell Neurosci.

## 4. Analysis of Results

### 4.1. Analysis of Bidirectional Short- and Long-Term Memory Networks

The introduction of an attention mechanism can control the influence of elements in the input sequence on the elements of the output sequence and retain more important information; based on the CNN-BO and LSTM-BO models, the *M* value is selected from 0.1 to 1.0, increasing by 0.1, respectively. The experimental results are shown in Figure 2. The accuracy of the two models increases and then decreases with the value of N. The accuracy of the LSTM-BO model is 82.25% and that of the CNN-BO model is 88.74% at *M* = 0.5, which are both the maximum values. The loss rate of the two models shows a general trend of decreasing and then increasing with the increase of *M* value, and at *M* = 0.5, the loss rate of the LSTM-BO model is 0.237 and the loss rate of the CNN-BO model is 0.167, which are both the minimum values. The above experimental results are analyzed, and the threshold *M* of the two models in this paper is taken as 0.6.

Dropout is an optimization method proposed to solve the overfitting and gradient disappearance problems of deep neural networks. To investigate the effect of dropout on the training results, this experiment takes the value of dropout from 0.1 to 1.0 and increases it by 0.1 in order, and the experimental results are shown in Figure 3. The highest accuracy of the LSTM-BO model is 79.86%, the lowest loss rate is 0.237, and the lowest time consumption is when the dropout is set to 0.2. The highest accuracy of the CNN-BO model is 87.75%.

### 4.2. Intelligent Computing IoT Model Analysis

The accuracy and F-value of the intelligent computing IoT model in the training process are shown in Figure 4, where Acc, measure, and loss in Figure 4 denote the accuracy and F-value of the training set in the training process, and val_acc and val_fmeasure denote the accuracy and F-value of the validation set in the training process, respectively. From Figure 4, it can be seen that, after 50 layers of iterations, the change curves of the four indicators have leveled off, indicating that the model in this chapter has reached the best training effect; from Figure 4, it can be seen that, after 50 layers of iterations, the loss in training has been reduced to the lowest level, indicating that the training goal of the intelligent computing IoT model has been achieved.

The article "A Study of Two-Way Short- and Long-Term Memory Network Intelligent Computing IoT Model-Assisted Home Education Attention Mechanism" was published in 2021. Journal: Comput Intell Neurosci.

The final experimental results of the four groups of models are shown in Figure 5. From the data in Figure 4, it can be seen that the algorithm model proposed in this chapter works best, and compared with the traditional CNN model, the accuracy of this algorithm increases from 87.63% to 92.51%, and the F-value increases from 87.92% to 93.22%, while its algorithmic performance far exceeds that of the SVM algorithm, which performs relatively well among the traditional machine learning algorithms.

### 4.3. Evaluation Analysis of Family Education Attention Mechanism

We converted the performance depicted by the ROC curve into a single scalar value by calculating the area under the ROC curve. Of course, the AUC serves as a more popular binary classifier evaluation metric, where a larger AUC value indicates better performance in the prediction of family education attention mechanisms. In Figure 6, the blue curve is generated from the first layer of the family education attention mechanism prediction, while the red curve is generated from the second layer of the family education attention mechanism prediction. The corresponding AUC values can also be seen in Figure 6. The AUC values for the predicted enhancer and enhancer strength categories are 0.934 and 0.842, respectively, and it is clear that, for identifying enhancers and nonenhancers, this AUC value is higher than the AUC value for the predicted enhancer strength category. However, both values reached a high level, which shows that the prediction of the family education attention mechanism we constructed has some accuracy and stability. When developing a classifier for predicting the attention mechanism of family education, the most important thing is to achieve the highest possible sensitivity while maintaining a low false alarm rate. The advantage of the ROC curve is that you can visualize all these performance indicators from a single image. Comparing the curve with the competitive model is a quick and easy way to choose the appropriate classification or diagnostic tool.

The dataset we used was of the same standard as the datasets of several other studies, and after we completed our prediction study to some extent, we compared the classification prediction results of various research methods to be able to analyze the effects of the study more objectively, and the results are shown in Figure 7. Comparing the Acc values of various family education attention mechanism predictions in the table, we can see that our constructed family education attention mechanism prediction iESW-2L2 is better than several existing family education attention mechanism predictions in identifying enhancers and nonenhancers, and the MCC value of the first layer of this family education attention mechanism prediction is the highest, indicating that this family education attention mechanism prediction has relatively good stability, and this paper's homeschooling attention mechanism prediction has generally improved in the first tier structure of the study. In addition, we can see from Figure 7 that the Acc value in the second layer of the family education attention mechanism prediction reaches 66.22%, which is second only to iEnhancerPred's 68.21% but has the best stability, indicating that the study has some effectiveness.

The article "A Study of Two-Way Short- and Long-Term Memory Network Intelligent Computing IoT Model-Assisted Home Education Attention Mechanism" was published in 2021. Journal: Comput Intell Neurosci.

## 5. Conclusion

Firstly, the current mainstream model deep neural network methods inside the field of artificial intelligence and big data research, forward propagation, and backward feedback methods in deep neural networks, classification of neural networks, and the structure and application of short- and long-term memory neural networks in recurrent neural networks are studied and analyzed. On this basis, the hidden layer activation function of the two-way recurrent neural network for short- and long-term memory is improved, and the improved neural network model is proposed in combination with the Morlet wavelet function. Based on simple discrete single-symbol text classification experiments, the effectiveness and performance of the model proposed in this paper are verified, by briefly elucidating the principles of the original recurrent neural network and the short- and long-term memory neural network and proposing the combination of the traditional wavelet function with the short- and long-term memory neural network, as well as changing the model levels and activation functions to improve the experimental results. The core goal of the attention mechanism is to quickly filter out high-value information from a large amount of data. The introduction of the attention mechanism in the homeschooling classification task can learn the dependencies within the court education and capture the internal structure of homeschooling. A two-way long- and short-term memory network intelligent computing IoT model to assist the attention mechanism of homeschooling is studied, a two-way long- and short-term memory network intelligent computing IoT model based on the two-way long- and short-term memory network is constructed, and its parameter modification rules of BP algorithm based on gradient descent are derived, respectively. To improve the recognition accuracy, a two-layer learning strategy is introduced, and the BP algorithm is used as the inner learning algorithm, while the outer learning adopts an improved particle swarm optimization algorithm, and the main innovation is to introduce the early convergence degree evaluation index to divide the population into three parts and adjust them adaptively to jump out of the local optimum, respectively. In this paper, we mainly study the sequence order information features by using various techniques to extract the sequence order information features. For feature extraction such as sequence structure, clustering algorithms, artificial intelligence analysis, and other methods can be used for in-depth research.

The article "A Study of Two-Way Short- and Long-Term Memory Network Intelligent Computing IoT Model-Assisted Home Education Attention Mechanism" was published in 2021. Journal: Comput Intell Neurosci.

## Figures and Tables

**Figure 1:** The characteristic model of family education attention mechanism.

**Figure 2:** Accuracy and loss rate variation.

**Figure 3:** Dropout selection experimental results.

**Figure 4:** Accuracy and F-value in training.

**Figure 5:** Experimental results.

**Figure 6:** The ROC plot of the predicted attention mechanism of family education.

**Figure 7:** Comparison of prediction results on the benchmark dataset.

**Table 1:** Model parameter configuration.

Serial number	Name	Meaning
1	Batch size	Number of batch training samples
2	Learning rate	E-learning efficiency
3	VALIDATION_SPLIT	The proportion of test set in training data set
4	Return sequences	Network return type
5	Early stopping	Model stop training parameters
6	NB epoch	Model iteration times

**Table 2:** Algorithm performance diagnosis description.

Serial number	AUC value range	Forecast description
1	AUC < 0.5	Not in line with the real situation
2	0.5 ≤ AUC < 0.8	Low accuracy
3	0.8 ≤ AUC < 0.8	Precise
4	AUC ≥ 0.8	With high accuracy

## Data Availability

The data used to support the findings of this study are available from the corresponding author upon request.
